The article "Drought Assessment Based on Data Fusion and Deep Learning" was retracted in 2023. Reasons: signs of a paper mill; suspected computer-generated content; unreliable results or conclusions; concerns about the data.

# Drought Assessment Based on Data Fusion and Deep Learning

**DOI:** 10.1155/2022/4429286

**Published:** 2022-07-31

**Authors:** Yanling Li, Bingyu Wang, Yajie Gong

**Affiliations:** School of Mathematics and Statistics, North China University of Water Resources and Electric Power, Zhengzhou 450046, China

## Abstract

Drought is a major factor affecting the sustainable development of society and the economy. Research on drought assessment is of great significance for formulating drought emergency policies and drought risk early warning and enhancing the ability to withstand drought risks. Taking the Yellow River Basin as the object, this paper utilizes data fusion, copula function, entropy theory, and deep learning, fuses the features of meteorological drought and hydrological drought into a drought assessment index, and establishes a long short-term memory (LSTM) network for drought assessment, based on deep learning theory. The results show that (1) after extracting the features of meteorological drought and hydrological drought, the drought convergence index (DCI) built on the fused features by copula function can accurately reflect the start and duration of the drought; (2) the drought assessment indices were effectively screened by judging the causality of the drought system, using the transfer entropy; (3) drawing on the idea of deep learning, LSTM for drought assessment, which was established on DCI and the drought assessment factors, can accurately assess the drought risks of the Yellow River Basin.

## 1. Introduction

Drought is a common natural disaster, which is usually induced by the abnormal reduction of rainfall. With a high frequency, a wide range of influence, and a high degree of damage, drought poses a serious threat to agricultural production, economic development, and social stability [1]. Statistics show that drought has killed 11 million people around the world. In the twentieth century alone, more than 2 billion were affected by drought [2]. The damage of drought is far more serious than that of any other disaster. The economic loss of a drought ranges from 6 to 8 billion USD per year [1]. Drought has obviously affected people's normal production and life, so the study of drought assessment has become a common concern of researchers.

With global warming, drought occurs more frequently and in a wider range across the globe. In many countries and regions, drought brings far more damage than flood. According to the Sixth Assessment Report (AR6) of the United Nations (UN) Intergovernmental Panel on Climate Change (IPCC), from 2010 to 2019, human activities caused global surface temperature to rise by 0.8°C–1.3°C [3]. The temperature rise would increase the scale and severity of drought. To make matters worse, the mass construction of water utilization projects and soil retention projects alters the state of the underlying surface and changes the evaporation, infiltration, runoff yield, and concentration, as well as the speed of water resource circulation [4].

The standardized precipitation index (SPI) is proposed by the World Meteorological Organization (WMO) to monitor the severity of drought [5]. The index can be calculated simply from uncomplex input data, which are easy to acquire. Applicable to multiple timescales, the SPI can meet the needs of different regions and applications, laying the basis for monitoring drought at different timescales. As the research goes deeper, scholars were no longer satisfied with the assessment and monitoring of a single type of drought and came up with composite drought indices. For example, Wu et al. [6] constructed a drought index coupling rainfall and soil water through fuzzy cloud reasoning and proved the reliability of the index by historical drought evolution. Won et al. [7] combined the copula function with SPI and the evaporation demand drought index into a joint drought index and applied the index to monitor the drought situation of atmospheric water supply. By kernel entropy component analysis, Han et al. [8] built a composite drought index encompassing rainfall, runoff, evapotranspiration, and soil water content and found that the index is highly sensitive to mild drought.

The drought cannot be fully illustrated by a single drought index alone. Therefore, many scholars have proposed considerable works to construct a series comprehensive drought index that cover as many drought variables as possible [9]. Ren et al. [10] combined SPI, PDSI, and SPEI into comprehensive drought indices through fuzzy comprehensive evaluation. Maji and Kanrar [11] proposed a comprehensive drought index by principal component analysis (PCA). Yet the combined drought index based on the weighting method and the fuzzy combined method has certain subjectivity in weighting, and it is easy to cause errors, and the combined drought index based on the principal component analysis method combines related variables linearly and cannot reflect their nonlinear impact characteristics.

Based on data fusion, DCI combining meteorological and hydrological factors was constructed, meteorological and hydrological drought for the feature layer fusion by copula function. Copula function is simply a specification of how univariate marginal distributions combine to form multivariate distribution. There is no limitation in choosing the marginal distribution function, and all margin-free characteristics can be fully maintained. The DCI not only has the characteristics of the meteorological drought index that can quickly capture the onset of drought but also has the advantage of the hydrological drought index that can describe the duration of drought, fusing meteorological and hydrological characteristics. The original information can be optimized and combined through data fusion, making it possible to turn multisource information into effective output. This paper extracts the features of hydrological drought and meteorological drought from the data collected at six major hydrological stations and meteorological stations along the trunk of the Yellow River and fuses the features with copula function, producing a hybrid drought index composed of both hydrological and meteorological factors. When selecting the drought factors, the influence between variables is measured by transfer entropy, and through this influence, a causal relationship between variables is established. Moreover, the LSTM network, a deep learning model, was adopted to evaluate drought by drought factors.

## 2. Study Area and Data Sources

The 5,464 km-long Yellow River (Figure 1) is the sixth longest in the world, and the second longest river in China, flowing through 9 provinces. The basin of the river, covering an area of 795,000 km^2^, spans across four geomorphic units: the Qinghai-Tibet Plateau, Inner Mongolia Plateau, the Loess Plateau, and North China Plain. Since the 1980s, the temperature rose significantly in the Yellow River Basin, while the rainfall dropped slightly [12]. Since the 1990s, the basin was hit by increasingly serious droughts. In 2009, a wide and severe drought plagued the Central Plains region, ringing a bell of the severity of drought [13]. In fact, the Yellow River Basin is the largest drought-stricken basin in China [14]. Drought has brought multiple problems, such as dried rivers and soil degradation [15]. It is of realistic significance to study the drought assessment of the Yellow River Basin, which would aid ecological balance and social development.

This paper selects the measured monthly runoffs of 1980–2019 at six major hydrological stations and the monthly meteorological data of 1980–2019 at 21 meteorological stations along the trunk of the Yellow River. On this basis, the meteorological and hydrological drought features were fused for assessment. The meteorological data were obtained from China Meteorological Data Service Center (http://data.cma.cn), and the hydrological data were collected from the official site of the Yellow River Conservancy Commission of the Chinese Ministry of Water Resources (http://www.yrcc.gov.cn/).

## 3. Methodology

### 3.1. Data Fusion

#### 3.1.1. Selection of Characteristic Parameters

The effectiveness of the copula function comes from the fact that the function can merge random marginal distributions, which contain the information of all variables, into a joint distribution, without losing or distorting any information. In 1993, McKee created SPI [16], a multitimescale drought index. The SPI can effectively assess the features of drought on different scales, using the occurrence probability of precipitation. The standardized runoff index (SRI) measures hydrological drought by river runoff and its statistic. The calculation process of the SRI is similar to that of the SPI [17, 18]. The drought/flood grading standards of SPI and SRI follow the *Grades of meteorological drought* (GB/T20481-2017), which was formulated by National Technical Committee on the Standardization of Climate and Climate Change of China.

#### 3.1.2. Copula Function

According to Sklar's theorem [19, 20], for any two one-dimensional (1D) random variables *X* and *Y*, if their distribution functions are *F*_*X*_(*x*) = *P*(*X* ≤ *x*) and *F*_*Y*_(*y*) = *P*(*Y* ≤ *y*), and their joint distribution function is *F*_*C*_(*x*,*y*), then there exists a unique copula function C() satisfying the following equation:

(1) $$\begin{array}{c} F_{C}\left(x,y\right)=C\left[F_{X}\left(x\right),F_{Y}\left(y\right)\right],x,y\in R. \end{array}$$

For two-dimensional (2D) variables, the common forms of copula function include Gaussian, Archimedean, and student T. Among them, the Archimedean copula is widely applied because it can reflect the dependence intensity with a parameter. The Archimedean copula can be further divided into three types: Gumbel, Clayton, and Frank. With asymmetric structures, Gumbel and Clayton copulas can capture the asymmetric properties. With a symmetric dependence structure, the Frank copula permits negative dependence by histogram of variables *X* and *Y*. The density function can be defined as

(2) $$\begin{array}{c} c^{Gu}\left(u,v;\theta \right)=\frac{C^{Gu}\left(u,v;\theta \right){\left(\ln\;u\cdot \;\ln\;v\right)}^{\theta -1}}{uv{\left[{\left(-\ln\;u\right)}^{\theta }+{\left(-\ln\;v\right)}^{\theta }\right]}^{2-1/\theta }}\left\{{\left[{\left(-\ln\;u\right)}^{\theta }+{\left(-\ln\;v\right)}^{\theta }\right]}^{1/\theta }+\theta -1\right\}, \end{array}$$

(3) $$\begin{array}{c} c^{Fr}\left(u,v;\theta \right)=\frac{-\theta \left(e^{-\theta }-1\right)e^{-\theta \left(u+v\right)}}{{\left[\left(e^{-\theta }-1\right)+\left(e^{-\theta u}-1\right)\left(e^{-\theta v}-1\right)\right]}^{2}}, \end{array}$$

(4) $$\begin{array}{c} c^{Cl}\left(u,v;\theta \right)=\left(1+\theta \right){\left(uv\right)}^{-\theta -1}{\left(u^{-\theta }+v^{-\theta }-1\right)}^{-2-1/\theta }, \end{array}$$

where *θ* is a parameter; *u* and *v* are marginal cumulative probabilities.

The parameter *θ* can be solved by the Kendall rank correlation coefficient *τ*. For the Gumbel copula, the relationship between *θ* and *τ* is *τ*=1 − 1/*θ*, *θ* ∈ [1, *∞*). For the Frank copula, that relationship is *τ*=1+4/*θ*(1/*θ*∫_0_^*θ*^*t*/*e*^*t*^ − 1*dt* − 1), *θ*∈*R/*{0}. For the Clayton copula, that relationship is *τ*=*θ*/*θ*+2, *θ* ∈ (0, *∞*).

For different objects, the fused feature between SPI and SRI can be described by the Euclidean distance between empirical copula function $\overset{\wedge }{C}\left(u,v\right)$ and copula function *C*(*u*, *v*) :

(5) $$\begin{array}{c} d=\sqrt{{\sum_{i=1}^{n}\left|C\left(u_{i},v_{i}\right)-\overset{\wedge }{C}\left(u_{i},v_{i}\right)\right|}^{2}}. \end{array}$$

The smaller the distance, the better the goodness-of-fit of copula function for the variables.

#### 3.1.3. Feature Layer Fusion

Let random variable *X* be the meteorological drought feature SPI, with a marginal distribution of *F*_*X*_(*x*). The joint distribution probability of drought features can be calculated by

(6) $$\begin{array}{c} F_{C}\left(x,y\right)=C\left[F_{X}\left(x\right),F_{Y}\left(y\right)\right]\\ =P\left(x\leq X,y\leq Y\right)\\ =p. \end{array}$$

The drought convergence index (DCI) can be expressed as

(7) $$\begin{array}{c} DC\;I=\varphi^{-1}\left(p\right), \end{array}$$

where *φ* is the standard normal distribution.

Referring to classification standards of SPI [21] and the National Climate Center's Standard, (GB/T20481-2017), droughts can be divided into different levels (Table 1) by severity.

According to the frequency of historical droughts and the empirical frequency of DCI, DCI = -1 was taken as the threshold of drought occurrence: if the DCI value remains below -1, the drought must have occurred.

### 3.2. Transfer Entropy

Considering the transmissibility between information, Schreiber [22] coined the concept of transfer entropy based on information entropy theory. Based on mutual information that reflects the correlation between variables, the transfer entropy measures the causality of information transfer in terms of magnitude and direction.

#### 3.2.1. Conditional Mutual Information

Conditional mutual information refers to the amount of mutual information acquired about event *y*_*j*_ based on the known event *x*_*i*_, under the given event *z*_*k*_:

(8) $$\begin{array}{c} I\left(y_{j};x_{i}|z_{k}\right)=\log\frac{p\left(y_{j}|x_{i},z_{k}\right)}{p\left(y_{j}|z_{k}\right)}. \end{array}$$

Solving the expectations of variables *X*, *Y*, and *Z*, the mean conditional mutual information of *X* relative to *Y* under *Z* can be obtained as follows:

(9) $$\begin{array}{c} I\left(Y;X|Z\right)=E\left[I\left(y_{j};x_{i}|z_{k}\right)\right]\\ =\sum_{j=1}^{N}\sum_{i=1}^{N}\sum_{k=1}^{N}p\left(y_{j},x_{i},z_{k}\right)\log\frac{p\left(y_{j}|x_{i},z_{k}\right)}{p\left(y_{j}|z_{k}\right)}\\ =\sum_{j=1}^{N}\sum_{i=1}^{N}\sum_{k=1}^{N}p\left(y_{j},x_{i},z_{k}\right)\log\;p\left(y_{j}|x_{i},z_{k}\right)-\sum_{j=1}^{N}\sum_{i=1}^{N}\sum_{k=1}^{N}p\left(y_{j},x_{i},z_{k}\right)\log\;p\left(y_{j}|z_{k}\right)\\ =H\left(Y|Z\right)-H\left(Y|X,Z\right). \end{array}$$

#### 3.2.2. Transfer Entropy

Suppose discrete variables *X*_*i*_ and *Y*_*i*_, *i* = 1, 2,…, *N* are of the same length and mutually act on each other. Then, the transfer entropy from *X* to *Y* reflects the information transfer from *X* to *Y* in the past states.

(10) $$\begin{array}{c} TE_{X⟶Y}=\sum P\left(Y_{i+1},X_{i},Y_{i}\right)\log\frac{P\left(Y_{i+1}|X_{i},Y_{i}\right)}{P\left(Y_{i+1}|Y_{i}\right)}\\ =\sum P\left(Y_{i+1},X_{i},Y_{i}\right)\log\;P\left(Y_{i+1}|X_{i},Y_{i}\right)-\sum P\left(Y_{i+1},X_{i},Y_{i}\right)\log\;P\left(Y_{i+1}|Y_{i}\right)\\ =H\left(Y_{i+1}|Y_{i}\right)-H\left(Y_{i+1}|X_{i},Y_{i}\right). \end{array}$$

According to the definition of transfer entropy, log *P*(*Y*_*i*_ _+_ _1_|*Y*_*i*_) is the occurrence probability of *Y*_*i*+1_ under the condition of state *Y*_*i*_, which excludes the influence of the past state of *Y* over its future information. In this way, *TE* can accurately measure the information transferred from *X* to *Y*. Conditional mutual information considers the dependence between variables *X* and *Y*, in the light of the information provided by variable *Z*. Transfer entropy considers the past state of variable *Y*, and the dependence between variables *X* and *Y*. Therefore, the following formula can be derived from the relationship between conditional mutual information and transfer entropy:

(11) $$\begin{array}{c} TE_{X⟶Y}=I\left(Y_{i+1};X_{i}|Y_{i}\right). \end{array}$$

### 3.3. Deep Learning

In deep learning, the recurrent neural network (RNN) has been widely and deeply applied in natural language processing (NLP), such as speech recognition, language modeling, and machine translation. The RNN has a good memory, supports parameter sharing, and realizes turing completeness. Therefore, it has lots of advantages in learning the nonlinear features of series.

Proposed by Hochreiter and Schmidhuber [23], the LSTM overcomes the defects of RNN by adding a memory unit to the recurrent layer, putting an end to the problem of exploding or vanishing gradients. The LSTM relies on the functions of the forget gate, the input gate, the output gate, and the memory unit to propagate and memorize long- and short-term information.  Figure 2 shows the structure of the LSTM.

During the operation of the LSTM, the forget gate firstly determines which information to forget in the current unit according to the input at the current state. The output state of the previous unit is controlled by the sigmoid function:

(12) $$\begin{array}{c} f_{t}=\sigma \left(W_{f}\left[h_{t-1},x_{t}\right]+b_{f}\right). \end{array}$$

The input gate consists of two parts. Firstly, the sigmoid layer determines which new information to add into the current unit. Then, the tanh layer obtains the new candidate state of the unit. Finally, the two are combined to obtain the state of the unit at the current moment *t*:

(13) $$\begin{array}{c} i_{t}=\sigma \left(W_{i}\left[h_{t-1},x_{t}\right]+b_{i}\right), \end{array}$$

(14) $$\begin{array}{c} {\tilde{C}}_{t}=\text{tanh}\left(W_{C}\left[h_{t-1},x_{t}\right]+b_{C}\right). \end{array}$$

The memory unit *C* stores the memory in the RNN and represents the long-term memory. The short-term memory is denoted by *h*. Both memories are propagated layer by layer backward to ensure the memory function of the LSTM:

(15) $$\begin{array}{c} C_{t}=f_{t}⊙C_{t-1}+i_{t}⊙{\tilde{C}}_{t}. \end{array}$$

From the past output, current input, and current unit state, the output gate drives the current output:

(16) $$\begin{array}{c} o_{t}=\sigma \left(W_{o}\left[h_{t-1},x_{t}\right]+b_{o}\right), \end{array}$$

(17) $$\begin{array}{c} h_{t}=o_{t}⊙\;\tanh\left(C_{t}\right), \end{array}$$

where *x*_*t*_ is the input of unit state; *f*_*t*_, *i*_*t*_, and *o*_*t*_ are the activation values of the forget gate, the input gate, and the output gate, respectively; ${\tilde{C}}_{t}$ and *C*_*t*_ are the candidate and output states, respectively; *h*_*t*_ is the output of the node; *W*_*f*_, *W*_*i*_, *W*_*c*_, and *W*_*o*_ are the weight matrices of the forget gate, the input gate, the unit state, and the output gate, respectively; *b*_*f*_, *b*_*i*_, *b*_*c*_, and *b*_*o*_ are the biases of the forget gate, the input gate, the unit state, and the output gate, respectively. The LSTM network uses the error backpropagation algorithm to update the weights. The weight is divided into two parts, one part participates in the output of the previous neuron as *W*_*fh*_, *W*_*ih*_, *W*_*ch*_, and *W*_*oh*_, and the other part participates in the current input as *W*_*fx*_, *W*_*ix*_, *W*_*cx*_, and *W*_*ox*_. *L* is the loss function, and the error at the current moment *t* is defined as

(18) $$\begin{array}{c} \delta_{t}\overset{\text{def}}{=}\frac{\partial L}{\partial h_{t}}. \end{array}$$

The input to the neuron is

(19) $$\begin{array}{c} {\text{net}}_{f,t}=W_{f}\left[h_{t-1},x_{t}\right]+b_{f}=W_{fh}h_{t-1}+W_{fx}x_{t}+b_{f}, \end{array}$$

(20) $$\begin{array}{c} {\text{net}}_{i,t}=W_{i}\left[h_{t-1},x_{t}\right]+b_{i}=W_{ih}h_{t-1}+W_{ix}x_{t}+b_{i}, \end{array}$$

(21) $$\begin{array}{c} {\text{net}}_{\tilde{c}}{\;}_{,t}=W_{c}\left[h_{t-1},x_{t}\right]+b_{c}=W_{ch}h_{t-1}+W_{cx}x_{t}+b_{c}, \end{array}$$

(22) $$\begin{array}{c} {\text{net}}_{o,t}=W_{o}\left[h_{t-1},x_{t}\right]+b_{o}=W_{\text{oh}}h_{t-1}+W_{ox}x_{t}+b_{o}, \end{array}$$

(23) $$\begin{array}{c} \delta_{f,t}\overset{\text{def}}{=}\frac{\partial L}{\partial {\text{net}}_{f,t}}, \end{array}$$

(24) $$\begin{array}{c} \delta_{i,t}\overset{\text{def}}{=}\frac{\partial L}{\partial {\text{net}}_{i,t}}, \end{array}$$

(25) $$\begin{array}{c} \delta_{\tilde{c},t}\overset{\text{def}}{=}\frac{\partial L}{\partial {\text{net}}_{\tilde{c},t}}, \end{array}$$

(26) $$\begin{array}{c} \delta_{o,t}\overset{\text{def}}{=}\frac{\partial L}{\partial {\text{net}}_{o,t}}. \end{array}$$

The error at *t*-1 is

(27) $$\begin{array}{c} \delta_{t-1}=\frac{\partial L}{\partial h_{t-1}}=\frac{\partial L}{\partial h_{t}}\frac{\partial h_{t}}{\partial h_{t-1}}=\delta_{t}\frac{\partial h_{t}}{\partial h_{t-1}}. \end{array}$$

## 4. Case Study

### 4.1. Data Fusion

Data fusion intends to combine information in the best possible way to obtain more effective information. This paper adopts the data fusion to combine meteorological data and hydrological data and evaluate the drought level comprehensively. It is worth noting that the data fusion generally falls into three levels: data layer fusion, feature layer fusion, and decision layer fusion. The fusion by copula function is the feature layer fusion because SPI and SRI, two characteristic indices, are adopted, which reflect meteorological and hydrological droughts, respectively.

#### 4.1.1. Selection of Copula Function

Taking the Tangnaihai Station in the upper reaches of the Yellow River for example, the frequency histograms and 2D frequency diagrams of SPI and SRI are displayed in Figure 3, and the cumulative distribution and density function diagrams of the Gumbel copula are displayed in Figure 4.

The SPI and SRI values of the Tangnaihai Station concentrated in [−2, 2]. The SPI frequency distribution was higher in the middle than the two sides and symmetric to a certain extent. The SRI frequency distribution was very asymmetric: the left side was taller than the right side. Thus, the distribution feature can be illustrated well by the Gumbel copula, which has the shortest Euclidean distance. Using the Gumbel copula, the authors established the copula function of the hybrid drought index for the Tangnaihai Station:

(28) $$\begin{array}{c} C^{Gu}\left(u,v;\theta \right)=\text{exp}\left\{-{\left[{\left(-\text{ln}u\right)}^{1.6008}+{\left(-\text{ln}v\right)}^{1.6008}\right]}^{0.6247}\right\}, \end{array}$$

(29) $$\begin{array}{c} c^{Gu}\left(u,v;\theta \right)=\frac{C^{Gu}\left(u,v;\theta \right){\left(\text{ln}u\cdot \text{ln}v\right)}^{0.6008}}{uv{\left[{\left(-\text{ln}u\right)}^{1.6008}+{\left(-\text{ln}v\right)}^{\theta }\right]}^{1.3753}}\left\{{\left[{\left(-\text{ln}u\right)}^{1.6008}+{\left(-\text{ln}v\right)}^{1.6008}\right]}^{0.6247}+0.6008\right\}. \end{array}$$

By the principle of Euclidean distance, the type of copula function was selected for each station.  Table 2 shows the selection results and the relevant parameters.

#### 4.1.2. Comparison of Drought Indices

Considering the situation of long-term drought, this paper computes the interannual SPIs and SRIs and conducts the feature layer fusion of meteorological and hydrological droughts by copula function, producing a hybrid drought index coupling long-term meteorological and hydrological information. Taking the Tangnaihai Station for example, the interannual SPI, SRI, and DCI were compared (Figure 5).

The threshold of moderate drought was set to -1. Normally, drought begins when the drought index falls below -1 and ends when the index rises above -1. The drought occurrence directly depends on rainfall. If the rainfall is consistently abnormal for a period, it will affect the confluence between surface water and groundwater through the natural water circulation and thus impact the hydrological condition. The SPI responds sensitively to the moment of the drought occurrence, while the SRI can accurately determine the duration and end time of drought. As shown in Figure 5, the DCI trend was overall similar to the trends of SPI and SRI. The three indices were consistent. The drought start time recognized by the DCI was earlier than that recognized by the SRI, and roughly the same as that identified by the SPI. Besides, the DCI recognized the same end time of drought as the SRI. Therefore, the DCI combines the merits of the SPI and the SRI: The DCI can sensitively capture the start time of drought as the SPI, and effectively depict the drought duration. By fusing meteorological information with hydrological information, the DCI can characterize both meteorological and hydrological droughts simultaneously. The advantages of the DCI include high sensitivity, strong recognizability, and wide applicability. This research further validated the theory of Kimaru et al. [21] and meteorological drought occurs and terminates very quickly, while hydrological drought begins and ends with a certain delay in response to meteorological drought.

### 4.2. Selection of Assessment Factors

When selecting the drought factors, the influence between variables is measured by transfer entropy, and through this influence, a causal relationship between variables is established. Based on conditional mutual information, the transfer entropy is an asymmetric measure [24]. Let TEX⟶Y be the information transfer from *X* to Y; TEY⟶X be the information transfer from Y to *X*. If TEX⟶*Y* > TEY⟶X, the influence of *X* over Y is stronger than that of Y over *X*. Then, *X* would be regarded as a driver of Y. Then, two variables were defined as *Y* = {DCI12} and *X* = {Drought factors}.  Table 3 shows the values of TEX⟶Y and TEY⟶X.

Table 3 shows that TEX⟶*Y* < TEY⟶*X* held for rainfall, air pressure, and vapor pressure. Thus, these factors are largely constrained by drought and are not the causes of drought. In the long run, drought is mainly affected by constantly changing factors. The action of drought will affect the natural water circulation, thereby constraining the formation of clouds, rains, and fogs. As a result, meteorological factors like rainfall, and air pressure will be influenced by drought. Rainfall, as an instantaneous factor, drive short-term drought more significantly than long-term drought. Drought will be influenced only if the rainfall increases or decreases continuously and breaks the balance of water circulation. Overall, this paper chooses the following factors to evaluate drought: air temperature, runoff, humidity, sunshine hours, and wind velocity.

### 4.3. LSTM Drought Evaluation Model

#### 4.3.1. Data Preprocessing

To speed up model training, min-max normalization was chosen to preprocess the data:

(30) $$\begin{array}{c} x_{i}^{*}=\frac{x_{i}-x_{\text{min}}}{x_{\text{max}}-x_{\text{min}}}, \end{array}$$

where *x*_*i*_ and *x*_*i*_^*∗*^ are the original data and the normalized data, respectively, and *x*_max_ and *x*_min_ are the maximum and minimum of the data, respectively.

#### 4.3.2. Model Training

To ensure the consistency between the data distribution of input and output variables, the first 90% of the original data were taken as the training set; the number of hidden layer nodes was set to 65; the batch size was set to 88; the number of iterations was set to 2,600; the mean squared error (MSE) was taken as the loss function. On this basis, an LSTM network was established. To prevent vanishing gradients, a rectified linear unit (ReLU) was selected as the activation function. The Adam optimizer was employed to optimize the model. Drawing on the features of momentum and root mean square propagation (RMSProp), adaptive learning rates were designed from parameters like the first and second order moment estimations of gradients, aiming to effectively update the weights.

#### 4.3.3. Model Evaluation

The model performance was evaluated by MSE and *R*^2^. The evaluation results are listed in Table 4.

As shown in Figure 6 and Table 3, the LSTM network can accurately assess the drought risks. The MSE was always smaller than 0.0032 and minimized at 0.0015. The *R*^2^ was always greater than 0.96, peaking at 0.9934. The interannual drought fluctuation was gentle, and the drought occurrence probability was low and highly predictable. Thus, the LSTM achieved a high prediction accuracy with a strong stability.

#### 4.3.4. Drought Assessment

Using the meteorological and hydrological data of 1980–2019, the multivariate LSTM network was called to assess the drought risks. As shown in Figure 7, the upper reaches of the Yellow River would be humid, the lower reaches would be normal, and the middle reaches would be dry in 2020. The prediction agrees with the actual situation in 2020.

Inspired by the working mode of the human brain, deep learning analyzes and learns the data by an artificial neural network (ANN) with multiple deep layers, which mimics the human brain. The long short-term memory (LSTM) network, as a deep learning neural network, can extract abstract, representative features from the original data. Capable of sequential and directional circulation, the LSTM is very suitable for analyzing the correlated time series. Poornima and Pushpalatha [25] found that the LSTM outperformed the autoregressive integrated moving average (ARIMA), and improved the prediction accuracy of the LSTM by adding humidity and temperature to training, both of which are positively correlated with the drought index. Dikshit et al. [26] achieved a high prediction accuracy with the LSTM neural network. Wu et al. [27] described monthly rainfall with wavelet transform, ARIMA, and LSTM, and demonstrated that the proposed W-A-L composite model can predict rainfall accurately, providing a good reference for further research into drought prediction.

## 5. Conclusions

The Yellow River Basin is frequently hit by drought, owing to the complex natural conditions, unique climate features, and special geographical conditions. The drought index and evaluation are important issues in the understanding and prevention of drought. Taking rainfall and runoff as meteorological and hydrological factors, this paper explores the nonlinear relationship between meteorological and hydrological series by the copula function, and constructs a hybrid drought index through the feature layer fusion. Then, the transfer entropy was computed for drought factors and indices, the causality was judged by the direction of information flow, and multiple factors were chosen for drought assessment. Further, the data information was mined through deep learning and used to build a multivariate LSTM network for drought evaluation. The main conclusions are as follows:

1. Following the idea of copula function, the hybrid drought index DCI combines the features of rainfall and runoff, and integrates the merits of SPI and SRI. The index can detect the drought occurrence as the SPI, and capture the drought duration as the SRI, providing an effective tool to depict the start, end, and progression of drought.
2. The transfer entropy was adopted to analyze the causality between climate and hydrological factors and the drought index, and judge the direction of information flow. In this way, the air temperature, runoff, humidity, sunshine hours, and wind velocity were selected to assess the interannual drought in the Yellow River Basin.
3. A deep learning model was established for drought assessment. The assessment accuracy of the LSTM network was proved by comparing the predicted values with the actual values, and by computing the evaluation metrics.

Drought research is a hot field among researchers. More scientific studies are expected for the driving mechanism, evolution, and evaluation of drought. In the era of the big data, data fusion and deep learning could be combined to open a bright new arena of drought research.

## Figures and Tables

**Figure 1:** Yellow River Basin.

**Figure 2:** Structure of the LSTM.

**Figure 3:** Histogram of SPI and SRI.

**Figure 4:** Cumulative distribution function and probability density function of the Gumbel copula.

**Figure 5:** Comparison of interannual drought indexes at the Tangnaihai Station.

**Figure 6:** Comparison of assessment effects of the LSTM model.

**Figure 7:** LSTM assessment of droughts for 2020.

**Table 1:** Division of drought levels.

DCI	Drought levels
(−∞,−2.0]	Extreme drought
(−2.0, −1.5]	Severe drought
(−1.5, −1.0]	Moderate drought
(−1.0, ∞)	No drought

**Table 2:** Copula functions for different stations.

Location	Station	Gaussian	T	Gumbel	Frank	Clayton	Selected function and parameter *θ*
Upper reaches	Tangnaihai	1.2443	1.2681	0.0490	0.1151	0.4732	Gumbel copula *θ* = 1.6008
	Shizuishan	3.6693	3.6773	0.0468	0.0548	0.0812	Gumbel copula *θ* = 1.0816

Middle reaches	Longmen	2.8618	2.8965	0.1403	0.0736	0.0639	Clayton copula *θ* = 0.4531
	Sanmenxia	2.3053	2.3308	0.0545	0.0603	0.0672	Gumbel copula *θ* = 1.2932

Lower reaches	Huayuankou	3.8682	3.8848	0.0619	0.0542	0.0617	Frank copula *θ* = 0.6412
	Lijin	3.9394	3.9606	0.1140	0.0959	0.0878	Clayton copula *θ* = 0.1540

**Table 3:** Transfer entropies between drought influencing factors and the drought index.

Location	Upper reaches		Middle reaches		Lower reaches	
Transfer entropy	TEX⟶Y	TEY⟶X	TEX⟶Y	TEY⟶X	TEX⟶Y	TEY⟶X
Air temperature	0.1414	0.0740	0.1590	0.1022	0.1555	0.1290
Runoff	0.1304	0.1034	0.1394	0.1222	0.1410	0.0880
Rainfall	0.1252	0.1633	0.1717	0.2066	0.1215	0.1947
Humidity	0.1525	0.1059	0.1731	0.1537	0.1790	0.1083
Air pressure	0.1026	0.1049	0.1663	0.1724	0.1535	0.1542
Vapor pressure	0.1412	0.1611	0.1564	0.1638	0.1540	0.1647
Sunshine hours	0.1740	0.1348	0.1494	0.1353	0.1418	0.0838
Wind velocity	0.1360	0.0714	0.1564	0.0874	0.1925	0.1204

**Table 4:** Evaluation index of the LSTM drought assessment model.

Evaluation index	Station					
	Tangnaihai	Shizuishan	Longmen	Sanmenxia	Huayuankou	Lijin
MSE	0.0015	0.0031	0.0028	0.0021	0.0019	0.0029
*R * ^2^	0.9602	0.9738	0.9917	0.9626	0.9639	0.9934

## Data Availability

The data used to support the findings of this study are available from the corresponding author upon request.
